The article "Adipose-Derived Stem Cell Exosomes Inhibit Hypertrophic Scaring Formation by Regulating Th17/Treg Cell Balance" was retracted in 2023. Reasons: signs of a paper mill; suspected computer-generated content; unreliable results or conclusions; lack of ethics approval or compliance.

# Adipose-Derived Stem Cell Exosomes Inhibit Hypertrophic Scaring Formation by Regulating Th17/Treg Cell Balance

**DOI:** 10.1155/2022/9899135

**Published:** 2022-10-12

**Authors:** Hongtao Wang, Yan Li, Zhang Yue, Yang Liu, Qiaohua Chen, Dahai Hu, Juntao Han

**Affiliations:** Department of Burns and Cutaneous Surgery, Xijing Hospital, Fourth Military Medical University, Xi'an 710032, China

## Abstract

Aiming to reveal the role of ADCS-Exos in secretion of inflammatory factors, Th17 and regulatory T (Treg) cell differentiation from naïve CD4+ T cells in hypertrophic scaring formation and maturation is explored. ELISA, qRT-PCR, and immunoblotting are performed to assay the local inflammatory factors IL-6, IL-10, IL-17A, and TNF-*α*, and transcriptional factors of ROR*ϒ*t and Foxp3, in scaring tissue from patients and mice wound models treated with or without ADCS-Exos. Immunohistochemistry staining and immunoblotting are conducted to assay the extracellular matrix (ECM) deposition in vitro and in vivo. The results show that IL-6, IL-10, IL-17A, TNF-*α*, ROR*ϒ*t, and Foxp3 are increased on mRNA and protein levels in hypertrophic scaring compared with atrophic scaring and normal skin. Naïve CD4^+^ T cells treated with ADCS-Exos in vitro can produce significantly less IL-6, IL-17A, TNF-*α*, and ROR*ϒ*t and more IL-10 and Foxp3 on mRNA and protein levels. In addition, mice in ADSC-Exos-treated group demonstrate less collagen deposition; decreased IL-17A, TNF-*α*, and ROR*ϒ*t; and increased IL-10 and Foxp3 production.

## 1. Introduction

Scaring is a consequence of abnormal wound healing when body tissues are damaged by a physical injury, such as burn, trauma, or surgery. In addition to itching and pain, scars can result in serious functional and cosmetic disability. The incidence rate ranges from 40% to 94% following surgery and from 30% to 91% following partial thickness burn injury [1]. Normal skin wound healing procedure involves inflammation, proliferation, and tissue remodeling [2]. Scaring regularly go through the remodeling processes of hyperplasia, stability, and atrophy (or called maturation), which last for 2–18 months after injury [3]. There are few effective therapies for prevention of scaring formation or promotion of scaring maturation, as the underlying mechanisms of hypertrophic scaring formation are poorly understood until now. Hypertrophic scaring is mainly characterized by hyperplasia of fibroblasts and disordered deposition of extracellular matrix (ECM). It is widely accepted that overproduction of inflammatory factors and persistent inflammation of the injured skin may play critical role in hypertrophic scaring formation [4]. The proinflammatory cytokines, such as IL-1, IL-6, IL-17A, and TNF-*α*, increase fibroblast proliferation and ECM production, as well as inhibit collagenase activity [5]. It was also indicated that anti-inflammatory therapy will be an effective strategy to avoid scaring formation or prompt scar maturation.

CD4^+^ T cells are crucial for directing appropriate immune responses for the pathogenesis of inflammatory diseases. When CD4^+^ T cells are activated, they differentiate into several subsets of effector cells, including T helper (Th) cells, such as Th1, Th2, and Th17, and regulatory T (Treg) cells [6]. Among these subsets, Th17 cells are unique proinflammatory cells characterized by transcriptional factor ROR*γ*t and cytokine IL-17A [7, 8]. Several studies have found that Th17 cells triggered persistent and uncontrolled inflammation in the pathogenesis of many human autoimmune diseases [9]. Alternatively, Treg cells inhibit recruitment and differentiation of inflammatory cells to maintain immune homeostasis by producing anti-inflammatory cytokines IL-10 [10, 11]. Thus, Th17 and Treg cells conduct opposite function during inflammatory and immune responses, and an inflammatory environment controls the balance between Treg and Th17 cells differentiation [12]. As result, impaired balance between Th17 and Treg cells has been recently implicated in various autoimmune disorders, as well as development of fibrosis in both patients and animal models [13, 14]. Nevertheless, whether Th17/Treg cell imbalance participates the formation and maturation of scaring is unintelligible, and it is of key importance to identify novel strategies to modulate balance of Th17/Treg cells. Several studies have confirmed that adipose-derived stem cells (ADSCs) participated in immune regulation and controlled inflammatory or autoimmune diseases, including enteritis, osteoarthritis, systemic sclerosis, idiopathic pneumonia, chronic liver fibrosis, renal fibrosis, and other diseases [15]. Moreover, ADSCs are expected to reduce inflammation, stimulate angiogenesis, promote wound healing, and inhibit abnormal scaring formation by secreting different bioactive substances [16–18]. However, stem cell therapy has several drawbacks, such as potential tumorigenesis, nonspecific differentiation, and the difficulty of quality control before administration. As result, to date, there is no clinical evidence for the use of ADSCs in the treatment of a hypertrophic scaring [19]. Recent studies revealed that ADSCs reduce inflammation mainly by paracrine secretion. Growing evidences suggest that exosomes (Exos), which contain information regulation between stem cells and target cells, could be a promising alternative to cell-based therapy [20]. ADSC-Exos are nanovesicles (30–150 nm) and can easily circulate through the body and reach areas of injury, and not toxic after repeated administration over long periods of time [21]. As result, ADSC-Exos are a promising therapeutic agent with immunomodulation and antifibrosis activity. Our previous study demonstrated that the levels of Th17 and its cytokine IL17A were significantly increased in hypertrophic scaring compared with normal skin [22]. Further, we illustrated that ADSC-Exos attenuated the deposition of collagen in hypertrophic scaring by inhibiting IL-17RA/Smad2/3 axis in vitro and in vivo [23].

In this study, we examine the effects of ADSC-Exos on Th17 and Treg cell differentiation and their related cytokines in vitro and in vivo to clarify whether ADSC-Exos can rectify the impaired Th17/Treg balance in hypertrophic scaring.

## 2. Related Work

Hypertrophic scaring is characterized by overproliferation of fibroblast and excessive deposition of ECM [24]. Inflammatory cells, as well as proinflammatory and anti-inflammatory cytokines, play critical role in the formation and maturation of scaring [25, 26]. Especially in the early stage of scaring formation, many inflammatory cells, such as neutrophils, mast cells, macrophages, and T lymphocytes, infiltrate into the tissue and regulate or secrete numerous proinflammatory factors, including IL-1, IL-6, and TNF-*α* [27, 28]. Specific cytokine in the immune system could activate naïve CD4^+^ T cells to differentiate into different T cell subsets, including proinflammatory Th17 and anti-inflammatory Treg [29]. Elevated IL-6 and TNF-*α* promoted naïve T cells to differentiate into Th17 cells, creating an enriched proinflammatory cytokine IL-17A [30]. Th17 cells are a group of CD4^+^ T lymphocyte subset regulated by specific transcription factor ROR*ϒ*t, while Treg cells mediate the inhibition of autoimmunity with Foxp3 and IL-10 as differentiation markers [31–33]. The imbalance of Th17/Treg cells leads to dysregulated immune responses such as autoimmune/inflammatory diseases [34, 35]. However, limited information is known about the local balance of Th17/Treg cells in hypertrophic scaring formation or maturation due to the difficulties in isolation T cells from scaring [36, 37].

IL-10 is considered attenuation of fibrosis by downregulating the collagen expression in fibroblasts [38]. IL-10 should be downregulated in the hypertrophic scaring as well as FoxP3 [39]. An overabundance of regulatory cell types may participate the formation and maturation of scaring. However, the ratio of ROR*γ*t/Foxp3, presenting the ratio of Th17/Treg, was increased in hypertrophic scaring compared with atrophic scaring and normal skin, revealing that augmented ratio of Th17/Treg may facilitate the formation of hypertrophic scaring. It is widely recognized that several cytokines and microRNAs affect the balance between Th17 and Treg [40]. Exploring the specific factors involved in the differentiation of naïve CD4^+^ T cells is promising effective strategies to inhibit hypertrophic scaring formation or prompt scaring maturation. Recently, several studies have demonstrated that ADSCs can be recruited to inflammatory or injury sites [41, 42], regulating inflammatory cells and cytokines and reprograming the inflammatory response. These properties make ADSCs a promising therapeutic intervention for autoimmune or inflammatory diseases [43]. ADSCs have been suggested as an alternative to immunosuppression in enteritis, osteoarthritis, systemic sclerosis, idiopathic pneumonia, chronic liver fibrosis, and renal fibrosis, as well as in tissue regeneration and healing [44]. It was revealed that ADSCs facilitate the proliferation and migration of fibroblasts in the early stages of wound healing and inhibit fibroblast proliferation and collagen synthesis in the late stage [45, 46]. Hence, ADSCs play different roles regulating wound healing and scar formation [47]. ADSCs can modulate both innate and adaptive immune responses acting on several types of immune cells through exchanging cytoplasmic components bidirectional with primary T lymphocytes [48]. In vitro, one of the hallmarks of ADSC immunomodulatory activity is the suppression of Th and upregulation of Treg [49].

ADSC-mediated effects on T cells proliferation and differentiation depend on several mechanisms, including cell-to-cell contact and secretion of soluble factors [50, 51]. Accumulated evidence has proved that ADSC-Exos, carrying complex biological information, including mRNAs, microRNAs (miRNAs), and soluble proteins, interact with target cells and influence their fate in tissue regeneration and remolding [52, 53]. It was documented in clinical or animal models that ADSC-Exos protect against cardiac, lung, liver, and kidney injuries, which is largely due to their anti-inflammatory, antiapoptotic, and proangiogenetic effects [54]. ADSC-Exos demonstrated the ability to inhibit T cell proliferation and differentiation, decrease the release of proinflammatory cytokines, and coordinate the balance between various subsets of CD4^+^ T cells [55, 56]. However, whether ADSCs-Exos are involved in the regulation of Th17/Treg cells in scaring formation and maturation needs further analysis. Our lab indicated that ADSC-Exos inhibit the proliferation of HSFs and reduce the deposition of ECM by inhibiting activation of IL-17RA/p-Smad2/3 axis. Moreover, a faster wound healing and less scar formation were observed in the mice treated with ADSC-Exos. The experiments in vivo further revealed that ADSCs-Exos downregulated the ECM deposition by regulating the inflammatory reaction and ratio of Th17/Treg cells. Meanwhile, reduced functionality of Treg cells is associated with upregulation of ROR*γ*t [57]. It is important to conduct comprehensive evaluation of how the ADSCs-Exos influence balance of Th17/Treg cells may play a part in new therapies in scaring formation.

## 3. Materials and Methods

### 3.1. Tissue Collection and Ethics

Postburn hypertrophic scaring, atrophic scaring, normal skin, and adipose tissues are collected from patients who underwent scaring excision and full thickness skin allograft reconstruction surgery in our department (Xi'an, China). All patients are informed of the purpose of the study and agreed to offer their excised tissues. The study is approved by the Ethics Committee of Xijing Hospital, Fourth Military Medical University.

### 3.2. Identification and Collection of ADSC-Exos

Human subcutaneous adipose tissues are trimmed and digested by 1 mg/mL collagenase type I (Gibco, USA) at 37°C for 60 min [23]. After centrifugation at 1000 × g for 5 min, the cell-debris pellet is resuspended in human ADSC Expansion Media (OriCell medium, China). Cell-conditioned medium is collected from 70 to 90% confluent ADSCs at 3–5 passages [58]. Differential ultracentrifugation at 4°C is used to separate the Exos from the collected medium [24]. Firstly, the supernatants are centrifuged at 300×*g* for 10 min and then at 2,000×*g* for 10 min to remove debris and dead cells. After centrifugation at 10,000×*g* for 30 min, the supernatant is ultracentrifuged at 100,000×*g* for 70 min using a Ti70 rotor (Optima XPN-100 Ultracentrifuge, USA). The morphology of Exos is observed by transmission electron microscope (TEM), and the particle size distribution is analyzed by nanoparticle tracking analysis (NTA). Exosomal markers CD9 and CD63 are determined by immunoblotting.

### 3.3. Isolation of Naïve CD4+ T Cells

The naïve CD4+ T cells is isolated and cultured as followed [25]. Spleens are harvested from 6 to 8 weeks C57BL/6 mice, and single cell suspension is obtained by smashing with a syringe plunger on sterile nylon mesh. After centrifuging at 300×*g* for 5 min, cell pellet is resuspended with 2 mL red blood cell lysis buffer ACK (ammonium-chloride-potassium) for 90 s. Then, a magnetic cell sorting method is used to isolate CD4+ T lymphocytes following the manufacturer's instructions (Invitrogen, USA). CD4+ T cells are then cultured in complete RPMI (Gibco, Paisley, UK). After 24-h starvation, cells are treated with ADSC-Exos at low concentration (10 *μ*g/mL), middle concentration (20 *μ*g/mL), and high concentration (40 *μ*g/mL), or are left untreated (as negative controls) for another 24 h. Then, the cytokines and transcriptional factors are assayed by ELISA, qRT-PCR, and immunoblotting.

### 3.4. The Isolation and Culture of Hypertrophic Scaring Fibroblasts (HSFs)

Tissue block explant is used to isolate HSFs as previously described [11]. HSFs between 3 and 5 subpassages are starved overnight when grown to 70–80% confluent and then cocultured with medium from CD4^+^ T cells or medium from CD4^+^ T cells pretreated with ADSC-Exos (20 *μ*g/mL) for 24 h. Then, the mediums are collected for ELISA, and cell lysates are used to RT-PCR or immunoblotting staining assay.

### 3.5. In Vivo Experiment

Male C57BL/6 mice (6-8 weeks old) are purchased from the Experimental Animal Center of Fourth Military Medical University. The mice are divided into two groups randomly: PBS or ADSC-Exos groups. A 1 × 1 cm^2^ full-thickness defects are created on the dorsal skin of the mice after anesthesia by isoflurane. From day 3 postoperation, ADSC-Exos or an equal volume of PBS is injected subcutaneously into the wound for the consecutive 5 days. Mice are sacrificed after 2 weeks when the wound healed, and wound tissues are harvested for further assays.

### 3.6. Histopathology Analysis

Scaring tissues from patients or mice are fixed, dehydrated, embedded, and cut according to conventional methods. Hematoxylin and eosin (H&E) and Masson's trichrome staining are conducted to observe histological change and ECM deposition. For immunohistochemistry staining, the slides are incubated with the primary antibodies against col I (1 : 100, Abcam, UK), col III (1 : 100, Abcam, UK), and *α*-SMA (1 : 200, Abcam, UK) overnight at 4°C. Next, the slides are incubated with biotinylated antibody (Histostain™ kit, ZSGB, China) for 10 min at room temperature and visualized with diaminobenzidine (ZSGB, China). The slides are examined by FSX100 Bio Imaging Navigator (Olympus, Japan).

### 3.7. Immunofluorescence Staining of HSFs

HSFs are seeded on a 14-mm glass diameter, which are placed on 35-mm culture dishes. When cultured to approximately 50% confluence, HSFs are cocultured with medium from CD4^+^ T cells or CD4+ T cells pretreated with ADSC-Exo (20 *μ*g/mL) for 24 h. After the treatment for another 24 h, the glass diameters are fixed, permeated, and blocked. Primary antibodies (*α*-SMA, 1 : 200, Abcam, UK) are incubated overnight at 4°C. Next, secondary FITC antirabbit antibodies (1 : 200 Boster, China) are incubated on HSFs for 1 h at 37°C and counterstained with DAPI. An Olympus FSX100 microscope is used to observe the images.

### 3.8. Analysis of Cytokine Production by ELISA

Tissue supernatants or cell culture supernatant are collected, and the levels of IL-6, IL-10, IL-17A, and TNF-*α* are analyzed using DuoSet ELISA kit (R&D Systems, Germany) following the manufacturer's protocol. The concentration cytokines are calculated according to the appropriate standard curve.

### 3.9. Quantitative Real-Time Polymerase Chain Reaction (qRTPCR)

The total RNA is extracted from tissue or cell lines using TRIzol reagent (Takara, Japan) and quantified to confirm the concentration. About 500 ng of total RNA is reverse-transcribed into cDNA using Prime Script™ RT reagent kit (Takara, Japan). The cDNA is amplified with Ultra SYBR Mixture (CWBIO, China) and specific primers by Bio-Rad IQ5 Real-Time System (Bio-Rad, USA). The relative expression of target genes is calculated using 2 − *ΔΔ*CT method.

### 3.10. Western Blotting

The total protein is extracted from tissue or cells for 30 min with 50 mL lysis buffer (RIPA, Beyotime) containing 0.5 mL protease inhibitors (PMSF, Boster, China). The total protein concentration is quantified by BCA kit. Primary antibodies against to col I (1 : 1000, Abcam, UK), col III (1 : 1000, Abcam, UK), *α*-SMA (1: 1000, CST, USA), CD9, CD63 (1 : 1000, Proteintech, China), IL-6 (1 : 1000, Boster, China), IL-17A (1 : 1000, Boster, China), TNF-*α* (1 : 1000, Boster, China), IL-10 (1 : 1000, Abcam), TNF-*α* (1 : 1000, Boster, China), ROR*ϒ*t (1 : 1000, Boster, China) and Foxp (1 : 1000, Boster, China), and GAPDH (1 : 1000, Zhuangzhi, China) are used for the analysis. The intensity of protein expression and normalized against GAPDH is analyzed by ImageJ software.

## 4. Results and Analysis

### 4.1. Inflammatory Factors and T Lymphocytes Participated in Hypertrophic Scaring Formation and Maturation

We collected human postburn hypertrophic scaring, atrophic scaring, and normal skins samples and examined the deposition of ECM and production of inflammatory factors. Pathological test, Masson staining, immunohistochemical staining, and Western blotting show that hypertrophic scaring has more deposition of col I, col III, and *α*-SMA compared with normal skin and atrophic scaring, as shown in Figure 1. The levels of proinflammatory cytokines (IL-6, IL-17A, and TNF-*α*) and anti-inflammatory cytokine (IL-10) are determined by ELISA, as shown in Figure 2. The results show that compared with normal skin and atrophic scaring, hypertrophic scaring produced much more IL-6, IL-17A, TNF-*α*, and IL-10. We failed to isolate Th17 and Treg cells in scaring tissue and normal skin because of limited cell numbers, and then, we checked the expression of ROR*ϒ*t and Foxp3, which are important transcriptional regulators of Th17 and Treg cells differentiation and function [26]. The results show that protein and mRNA levels of ROR*ϒ*t and Foxp3 in hypertrophic scaring are significantly higher than that of atrophic scaring and normal skin. However, the protein ratio of RORϒt/Foxp3 is 1.51 ± 0.28 in hypertrophic scaring, 0.84 ± 0.32 in atrophic scaring, and 0.70 ± 0.32 in normal skin. The difference is statistically significant, indicating that inflammatory factors and balance of Th17/Treg cells may participate in the formation and maturation of scaring.

### 4.2. ADSC-Exos Decreased the Production of Proinflammatory Factors by CD4+ T Cells and Promoted T Cells Differentiating into Treg Subset In Vitro

The results show that ADSC-Exos inhibited the deposition of extracellular matrix (ECM) and scaring formation in vitro and in vivo. To examine the role of ADSC-Exos in naïve CD4^+^ T cell differentiation, we collected Exos from medium of ADSCs. As shown in Figure 3(a), Exos is round, oval-shaped, and lipid bilayer membrane-bound structures. NTA identified the diameters of Exos are in a range of 100–150 nm, as shown in Figure 3(b) and Figure 3(c). Western blot results confirm the presence of known exosomal markers CD63 and CD9, as shown in Figure 3(d). We then treated naïve CD4^+^ T cells in vitro with low (10 *μ*g/mL), middle (20 *μ*g/mL), and high (40 *μ*g/mL) concentration of ADSC-Exos for 24 h. The production of inflammatory factors is assayed by ELISA, as shown in Figure 4(a). As shown in Figure 4(b) and Figure 4(c), inflammatory factors, as well as transcript factors ROR*ϒ*t and Foxp3, are assayed by qRT-PCR.  Figure 4(d) shows Western blot analysis of exosomal markers (CD9, and CD63). The results demonstrate that the inflammatory IL-6, IL-17A, and TNF-*α* level is decreased in the CD4^+^ T cells treated with ADSCs-Exos compared with control groups, but IL-10 is significantly increased in the CD4^+^ T treated with ADSC-Exos group. In addition, ADSC-Exos increased the Foxp3, but decreased RORϒt expression in naïve CD4^+^ T cells on both mRNA and protein levels.

### 4.3. Medium from CD4+ T Cells Pretreated with ADSC-Exos Decreased the Production of ECM by HSF In Vitro

To certify whether ADSC-Exos decrease ECM production of HSFs through regulating CD4^+^ T cells differentiation, we treat HSF with medium of CD4^+^ T cells or medium of CD4^+^ T cells pretreated with ADSC-Exos for 24 h. As shown in Figure 5(a) and Figure 5(b), IFC results show that, compared with medium of CD4^+^ T cells, HSFs incubate with medium of CD4^+^ T cells pretreated with ADSC-Exos decreased expression of *α*-SMA. Immunoblotting results indicate that the medium of CD4^+^ T cells pretreated with ADSC-Exos inhibited the expression of col I, col III, and *α*-SMA compared with medium from CD4^+^ T cells, as shown in Figure 5(c).

### 4.4. ADSC-Exos Attenuated Hypertrophic Scaring through Regulating Subset Differentiation of T Cells In Vivo

We further investigate whether ADSC-Exos attenuated hypertrophic scaring through regulating subset differentiation of T cells in vivo. According to histological analysis, the ADSC-Exos inhibits the proliferation of fibroblast and deposition of ECM, such as col I, col III, and *α*-SMA, as shown in Figure 6(a). Western blotting results indicate that ADSC-Exos-treated mice produced less col I, col III, and *α*-SMA compared with control group, as shown in Figure 6(b). The proinflammatory factors, IL-6, IL-17A, and TNF-*α* are lower in ADSC-Exos-treated group compared to the PBS group, but IL-10 is significantly higher in ADSC-Exos-treated group by ELISA assay, and the difference is statistically significant, as shown in Figure 6(c). From Figures 6(d) and 6(e), the results of qRT-PCR and Western blotting show that mRNA and protein levels of IL-6, IL-17A, and TNF-*α* are lower, and IL-10 is higher in the ADSC-Exos group compared with control groups. To investigate the effect of treatment with ADSC-Exos on the differentiation of Treg cells in scaring tissue in mice, we applied qRT-PCR and Western blotting to check the level of transcriptional regulators ROR*ϒ*t and Foxp3, mRNA and protein level of RORϒt is lower, and Foxp3 is higher in ADSC-Exos groups compared with control groups.

## 5. Conclusions

In this study, adipose-derived stem cells exosomes inhibit hypertrophic scaring formation by regulating Th17/Treg cell balance are explored. We collect human postburn hypertrophic scaring, atrophic scaring, and normal skin samples and examine the levels of inflammatory factors. Consistent with previous researches, our results indicate that both proinflammatory cytokines, such as IL-6, IL-17A, and TNF-*α*, and anti-inflammatory cytokine IL-10 are increased in hypertrophic scaring compared with atrophic scaring and normal skin. Also, the expression levels of transcription factors ROR*γ*t and Foxp3, which are, respectively, specific to Th17 and Treg, are in increased in hypertrophic scaring. The results can provide some suggestions on the interplay between ADCS-Exos and CD4+ T cells in hypertrophic scaring.

## Figures and Tables

**Figure 1:** The deposition of ECM in postburn hypertrophic scaring, atrophic scaring and normal skin: (a) HE, Masson, and HIS of col I, col III, and *α*-SMA; (b) Western blot staining; and (c) protein expression of col I, col II, and *α*-SMA.

**Figure 2:** Inflammatory factors and transcriptional factors production in hypertrophic scaring, atrophic scaring, and normal skin: (a) ELISA results; (b) qRTPCR; and (c) results of Western blot.

**Figure 3:** The identification of ADSC-Exo: (a) The morphology of ADSC-Exo observed by TEM; (b) the distribution of ADSC-Exo analyzed by NTA; (c) the size of ADSC-Exo analyzed by NTA; and (d) Western blot analysis of exosomal markers (CD9 and CD63).

**Figure 4:** ADSC-exos promoted the production of IL-10 and FOXP3 and decreased generation of IL17A and ROR*γ*t: (a) inflammatory factors production in CD4^+^T cells in response to ADSC-exos or control by ELISA; (b) mRNA levels of inflammatory factors in CD4^+^T cells treated with or without ADSC-exos; (c) protein levels of inflammatory factors in CD4^+^T cells treated or not with ADSC-exos; and (d) Western blot analysis of exosomal markers (CD9 and CD63).

**Figure 5:** ADSC-Exos downregulated proinflammatory factors and ECM expression and upregulated anti-inflammatory factor expression by CD4^+^ T cells in vitro: (a) immunofluorescence staining in HSFs stimulated with medium from CD4^+^ T cells or CD4^+^ T cells pretreated with ADSC-Exo; (b) qRT-PCR analysis of col I, col III, and *α*-SMA; and (c) immunobloting analysis of col I, col III, and *α*-SMA in HSFs stimulated with medium from CD4^+^ T cells or CD4^+^ T cells pretreated with ADSC-Exo.

**Figure 6:** The effect of ADSC-Exos on the excisional model of mice in vivo: (a) H&E and immunohistochemistry staining on day 14 postwounding in wound tissues treated with ADSC-Exos or PBS; (b) immunoblot analysis of col I, col III, and *α*-SMA in wound tissues of mice; (c) ELISA analysis of inflammatory factors and transcriptional factors in wound tissues of mice treated with ADSC-Exos or PBS; (d) qRT-PCR analysis of inflammatory factors and transcriptional factors in wound tissues; and (e) immunoblot analysis of inflammatory factors and transcriptional factors in wound tissues of mice.

## Data Availability

The simulation experiment data used to support the findings of this study are available from the corresponding author upon request.

## Abbreviations

ADSCs: Adipose-derived stem cells
ECM: Extracellular matrix
Exos: Exosomes
H&E: Hematoxylin and eosin
HSFs: Hypertrophic scaring fibroblasts
IL: Interleukin
miRNAs: microRNAs
MSCs: Mesenchymal stem cells
NTA: Nanoparticle tracking analysis
qRTPCR: Quantitative real-time polymerase chain reaction
TEM: Transmission electron microscope
Th: T helper
Treg: Regulatory T cell.

## References

[1] Bloemen M. C., Van der Veer W. M., Ulrich M. M., Van Zuijlen P. P., Niessen F. B., Middelkoop E. (2009). Prevention and curative management of hypertrophic scar formation. *Burns*.

[2] Leung M. F., Wang J. (2021). Minimax and bi-objective portfolio selection based on collaborative neurodynamic optimization. *IEEE Transactions on Neural Networks and Learning Systems*.

[3] Oliveira G. V., Chinkes D., Mitchell C., Oliveras G., Hawkins H. K., Herndon D. N. (2005). Objective assessment of burn scar vascularity, erythema, pliability, thickness, and planimetry. *Dermatologic Surgery*.

[4] Ogawa R. (2017). Keloid and hypertrophic scars are the result of chronic inflammation in the reticular dermis. *International Journal of Molecular Sciences*.

[5] He B., Wang Y., Shao N., Chang H., Cheng Y. (2015). Polymers modified with double-tailed fluorous compounds for efficient DNA and siRNA delivery. *Acta Biomaterialia*.

[6] Zhu J., Paul W. E. (2010). Peripheral CD4+ T-cell differentiation regulated by networks of cytokines and transcription factors. *Immunological Reviews*.

[7] Kamali A. N., Noorbakhsh S. M., Hamedifar H. (2019). A role for Th1-like Th17 cells in the pathogenesis of inflammatory and autoimmune disorders. *Molecular Immunology*.

[8] Cai C. W., Blasé J. R., Zhang X., Eickhoff C. S., Hoft D. F. (2016). Th17 cells are more protective than Th1 cells against the intracellular parasite Trypanosoma cruzi. *PLoS Pathogens*.

[9] Korn T., Bettelli E., Oukka M., Kuchroo V. K. (2009). IL-17 and Th17 cells. *Annual Review of Immunology*.

[10] Gładysz D., Krzywdzińska A., Hozyasz K. K. (2018). Immune abnormalities in autism spectrum disorder-could they hold promise for causative treatment?. *Molecular Neurobiology*.

[11] Shi J., Li J., Guan H. (2014). Anti-fibrotic actions of interleukin-10 against hypertrophic scarring by activation of PI3K/AKT and STAT3 signaling pathways in scar-forming fibroblasts. *PLoS One*.

[12] Littman D. R., Rudensky A. Y. (2010). Th17 and regulatory T cells in mediating and restraining inflammation. *Cell*.

[13] Murao N., Seino K., Hayashi T. (2014). Treg-enriched CD4+ T cells attenuate collagen synthesis in keloid fibroblasts. *Experimental Dermatology*.

[14] Frantz C., Auffray C., Avouac J., Allanore Y. (2018). Regulatory T cells in systemic sclerosis. *Frontiers in Immunology*.

[15] Bateman M. E., Strong A. L., Gimble J. M., Bunnell B. A. (2018). Concise review: using fat to fight disease: a systematic review of nonhomologous adipose-derived stromal/stem cell therapies. *Stem Cells*.

[16] Zarei F., Abbaszadeh A. (2018). Stem cell and skin rejuvenation. *Journal of Cosmetic and Laser Therapy*.

[17] Zhang Q., Liu L. N., Yong Q., Deng J. C., Cao W. G. (2015). Intralesional injection of adipose-derived stem cells reduces hypertrophic scarring in a rabbit ear model. *Stem Cell Research & Therapy*.

[18] Guisantes E., Fontdevila J., Rodríguez G. (2012). Autologous fat grafting for correction of unaesthetic scars. *Annals of Plastic Surgery*.

[19] Cai Y., Li J., Jia C., He Y., Deng C. (2020). Therapeutic applications of adipose cell-free derivatives: a review. *Stem Cell Research & Therapy*.

[20] Lou G., Chen Z., Zheng M., Liu Y. (2017). Mesenchymal stem cell-derived exosomes as a new therapeutic strategy for liver diseases. *Experimental & Molecular Medicine*.

[21] Mendt M., Kamerkar S., Sugimoto H. (2018). Generation and testing of clinical-grade exosomes for pancreatic cancer. *JCI Insight*.

[22] Zhang J., Qiao Q., Liu M. (2018). IL-17 promotes scar formation by inducing macrophage infiltration. *The American Journal of Pathology*.

[23] Li Y., Zhang J., Shi J. (2021). Exosomes derived from human adipose mesenchymal stem cells attenuate hypertrophic scar fibrosis by miR-192-5p/IL-17RA/Smad axis. *Stem Cell Research & Therapy*.

[24] Théry C., Amigorena S., Raposo G., Clayton A. (2006). Isolation and characterization of exosomes from cell culture supernatants and biological fluids. *Current Protocols in Cell Biology*.

[25] Yang W., Chen X., Hu H. (2020). CD4^+^ T-cell differentiation in vitro. *Methods in Molecular Biology*.

[26] Li M. O., Rudensky A. Y. (2016). T cell receptor signalling in the control of regulatory T cell differentiation and function. *Nature Reviews. Immunology*.

[27] Huang X. L., Wang Y. J., Yan J. W. (2015). Role of anti-inflammatory cytokines IL-4 and IL-13 in systemic sclerosis. *Inflammation Research*.

[28] Murdaca G., Spanò F., Contatore M., Guastalla A., Puppo F. (2014). Potential use of TNF-*α* inhibitors in systemic sclerosis. *Immunotherapy*.

[29] Wei B., Pei G. (2010). MicroRNAs: critical regulators in Th17 cells and players in diseases. *Cellular & Molecular Immunology*.

[30] Zhang Q., Yamaza T., Kelly A. P. (2019). Tumor-like stem cells derived from human keloid are governed by the inflammatory niche driven by IL-17/IL-6 axis. *PLoS One*.

[31] Zhao L., Qiu D. K., Ma X. (2010). Th17 cells: the emerging reciprocal partner of regulatory T cells in the liver. *Journal of Digestive Diseases*.

[32] Lee G. R. (2018). The balance of Th17 versus Treg cells in autoimmunity. *International Journal of Molecular Sciences*.

[33] Sabat R., Wolk K., Loyal L., Döcke W. D., Ghoreschi K. (2019). T cell pathology in skin inflammation. *Seminars in Immunopathology*.

[34] Noack M., Miossec P. (2014). Th17 and regulatory T cell balance in autoimmune and inflammatory diseases. *Autoimmunity Reviews*.

[35] Zhu X., Zhu J. (2020). CD4 T helper cell subsets and related human immunological disorders. *International Journal of Molecular Sciences*.

[36] Wang Z., Zhao W., Cao Y. (2020). The roles of inflammation in keloid and hypertrophic scars. *Frontiers in Immunology*.

[37] Leung M. F., Wang J. (2022). Cardinality-constrained portfolio selection based on collaborative neurodynamic optimization. *Neural Networks*.

[38] Shi J., Wan Y., Shi S. (2015). Expression, purification, and characterization of scar tissue neovasculature endothelial cell-targeted rhIL10 in Escherichia coli. *Applied Biochemistry and Biotechnology*.

[39] Sabat R., Grütz G., Warszawska K. (2010). Biology of interleukin-10. *Cytokine & Growth Factor Reviews*.

[40] Glocker E. O., Kotlarz D., Klein C., Shah N., Grimbacher B. (2011). IL-10 and IL-10 receptor defects in humans. *Annals of the New York Academy of Sciences*.

[41] Gnecchi M., Zhang Z., Ni A., Dzau V. J. (2008). Paracrine mechanisms in adult stem cell signaling and therapy. *Circulation Research*.

[42] Nawaz M., Fatima F., Vallabhaneni K. C. (2016). Extracellular vesicles: evolving factors in stem cell biology. *Stem Cells International*.

[43] Li P., Guo X. (2018). A review: therapeutic potential of adipose-derived stem cells in cutaneous wound healing and regeneration. *Stem Cell Research & Therapy*.

[44] Mazini L., Rochette L., Admou B., Amal S., Malka G. (2020). Hopes and limits of adipose-derived stem cells (ADSCs) and mesenchymal stem cells (MSCs) in wound healing. *International Journal of Molecular Sciences*.

[45] Huayllani M. T., Sarabia-Estrada R., Restrepo D. J. (2020). Adipose-derived stem cells in wound healing of full-thickness skin defects: a review of the literature. *Journal of Plastic Surgery and Hand Surgery*.

[46] Qiu H., Liu S., Wu K., Zhao R., Cao L., Wang H. (2020). Prospective application of exosomes derived from adipose-derived stem cells in skin wound healing: a review. *Journal of Cosmetic Dermatology*.

[47] Li C., Wei S., Xu Q., Sun Y., Ning X., Wang Z. (2022). Application of ADSCs and their exosomes in scar prevention. *Stem Cell Reviews and Reports*.

[48] Matula Z., Németh A., Lőrincz P. (2016). The role of extracellular vesicle and tunneling nanotube-mediated intercellular cross-talk between mesenchymal stem cells and human peripheral T cells. *Stem Cells and Development*.

[49] Gonzalez-Rey E., Gonzalez M. A., Varela N. (2010). Human adipose-derived mesenchymal stem cells reduce inflammatory and T cell responses and induce regulatory T cells in vitro in rheumatoid arthritis. *Annals of the Rheumatic Diseases*.

[50] Wise R. M., Harrison M., Sullivan B. N. (2020). Short-term rapamycin preconditioning diminishes therapeutic efficacy of human adipose-derived stem cells in a murine model of multiple sclerosis. *Cell*.

[51] Kuca-Warnawin E., Janicka I., Bonek K., Kontny E. (2021). Modulatory impact of adipose-derived mesenchymal stem cells of ankylosing spondylitis patients on T helper cell differentiation. *Cell*.

[52] Ranganath S. H., Levy O., Inamdar M. S., Karp J. M. (2012). Harnessing the mesenchymal stem cell secretome for the treatment of cardiovascular disease. *Cell Stem Cell*.

[53] Xu Y., Deng M., Cai Y. (2020). Cell-free fat extract increases dermal thickness by enhancing angiogenesis and extracellular matrix production in nude mice. *Aesthetic Surgery Journal*.

[54] Hong P., Yang H., Wu Y., Li K., Tang Z. (2019). The functions and clinical application potential of exosomes derived from adipose mesenchymal stem cells: a comprehensive review. *Stem Cell Research & Therapy*.

[55] Bolandi Z., Mokhberian N., Eftekhary M. (2020). Adipose derived mesenchymal stem cell exosomes loaded with miR-10a promote the differentiation of Th17 and Treg from naive CD4^+^ T cell. *Life Sciences*.

[56] Blazquez R., Sanchez-Margallo F. M., de la Rosa O. (2014). Immunomodulatory potential of human adipose mesenchymal stem cells derived exosomes on in vitro stimulated T cells. *Frontiers in Immunology*.

[57] Yu F., Sharma S., Edwards J., Feigenbaum L., Zhu J. (2015). Dynamic expression of transcription factors T-bet and GATA-3 by regulatory T cells maintains immunotolerance. *Nature Immunology*.

[58] Cao W., Wang X., Chen T. (2015). The expression of notch/notch ligand, IL-35, IL-17, and Th17/Treg in preeclampsia. *Disease Markers*.

